# The Survival and Prognosis Characteristics of Primary Esophageal Small-Cell Carcinoma

**DOI:** 10.1155/2022/5615009

**Published:** 2022-09-30

**Authors:** Jie Li, Xiangmei Zhang, Xinjian Xu, Qi Zhao, Qing Yang, Ming He, Xin Chen, Jidong Zhao

**Affiliations:** ^1^Department of Medical Affairs, Fourth Hospital of Hebei Medical University, Shijiazhuang 050011, China; ^2^Research Center, Fourth Hospital of Hebei Medical University, Shijiazhuang 050011, China; ^3^Hebei Provincial Key Laboratory of Tumor Microenvironment and Drug Resistance, Hebei Medical University, Shijiazhuang 050017, China; ^4^Department of Thoracic Surgery, Fourth Hospital of Hebei Medical University, Shijiazhuang 050011, China; ^5^Department of Clinical Laboratory, Fourth Hospital of Hebei Medical University, Shijiazhuang 050011, China

## Abstract

**Objective:**

To comprehensively explore the survival characteristics of primary esophageal small-cell carcinoma (PSCCE) and identify the main factors affecting the prognosis.

**Methods:**

The clinical and follow-up data of PSCCE patients admitted to the Fourth Hospital of Hebei Medical University from 2006 to 2010 were retrospectively analyzed. The primary endpoint was five-year survival. Survival curves were drawn using the Kaplan-Meier method, and log-rank test was used to compare the differences in survival rates among the groups. Cox regression models were used to analyze prognostic factors.

**Results:**

A total of 119 eligible patients were retrieved. Median survival was 27 months (3-100 months). Changes in overall survival (OS) in PSCCE patients were associated with TNM stage (*P* = 0.007), T stage (*P* = 0.049), and lymph node metastasis (*P* = 0.004). When TNM was in stage I-IIb, lymph node metastasis (*P* = 0.003) or combined adjuvant therapy (*P* = 0.004) was an independent factor affecting OS. Survival analysis showed that TNM staging had no predictive value for 5-year survival time or disease-free survival (DFS) of PSCCE (*P* > 0.05).

**Conclusion:**

TNM stage, T stage, and lymph node metastasis were related to the survival of patients. Negative lymph node metastasis and treatment are independent prognostic factors in PSCCE TNM stage I-IIb patients.

## 1. Introduction

Primary small-cell carcinoma of esophagus (PSCCE) is a rare invasive malignant tumor, which was first reported by McKeown in 1952 [1], and accounts for 0.4-2.8% in all esophageal cancers [2]. In China, it is most commonly located in the middle of the esophagus, while it is most often located in the lower part of the esophagus in western countries [3]. Due to the highly invasive and metastatic nature of PSCCE, most patients often have distant metastases at initial diagnosis resulting in a very poor prognosis [4]. Studies have shown that the median survival time (MST) of PSCCE is about 14 to 28 months, and the 5-year overall survival time (OS) is about 6.7%-18% [5–7]. Although survival in PSCCE patients has improved with advances in surgery, chemotherapy, and radiation therapy [6], due to its low incidence, studies with large numbers of participants are still lacking. This limits our knowledge of the pathological mechanisms and characteristics of PSCCE, and no optimal treatment regimen has yet been identified.

Imaging examination is of little significance for the diagnosis of PSCCE [8]. Pathology is the gold standard for the diagnosis of esophageal small-cell carcinoma, including simple small-cell carcinoma and mixed small-cell carcinoma. The most common method for preoperative diagnosis is gastroscopy, but gastroscopic biopsy tissue is small, and the components of small-cell carcinoma and other types of cancer are often mixed in the same tissue, so the success rate of preoperative diagnosis is low [9]. In addition, studies suggest that patients with PSCCE are prone to lymph node metastasis or even distant metastasis [10]. These realities have greatly increased the threat of this disease to the lives of patients and raised the risk of poor prognosis.

So far, the high-risk factors of PSCCE have not been specified, except for drinking and smoking history [11, 12]. This is not conducive to disease prevention and clinical treatment. On this basis, the clinical data of 119 patients with PSCCE admitted to our hospital were retrieved and analyzed. We summarized the survival characteristics of the disease and identified risk factors that may affect the prognosis of the disease.

## 2. Methods

### 2.1. Patient Data

By consulting electronic medical records, we retrospectively evaluated PSCCE patients who were treated surgically at the Fourth Hospital of Hebei Medical University between January 1, 2005 and December 31, 2012. The study was conducted in accordance with the Declaration of Helsinki (as revised in 2013). The study was approved by the hospital ethics committee. All patients have signed informed consent at admission.

### 2.2. Inclusion and Exclusion Criteria

The patients selected for this study must meet the following inclusion criteria: (1) esophagectomy, complete postoperative pathological report (tumor length, depth, upper and lower disability, degree of differentiation, pathological type, etc.), and the number of lymph nodes ≥ 16; (2) postoperative pathology showed small-cell carcinoma of the esophagus, and there was no mixed component of other malignant tumors; (3) postoperative adjuvant therapy data were complete. Patients who met the following conditions were excluded from the study: (1) suffering from other malignant tumors outside the esophagus at the same time or at an appropriate time, (2) receiving antitumor therapy before surgery, and (3) ending non-PSCCE-related deaths.

### 2.3. Tumor Staging

All patients were staged according to the 8th edition of the tumor (T), nodes (N), and metastases (M) (TNM) staging system of the American Joint Committee on Cancer (AJCC) [13]. Cases without regional lymph node metastasis were defined as N0, cases with one to three regional lymph node metastases were defined as N1, and cases with more than three regional lymph node metastases were defined as N2.

### 2.4. Follow-Up Principles

Follow-up within 2 years after operation, review chest and upper abdomen CT and esophagography every 3 (±1) months, to determine regional lymph nodes and anastomosis. Adjuvant chemotherapy was defined as receiving platinum-containing combined chemotherapy ≥ 1 time after surgery.

### 2.5. Statistical Analysis

Five-year survival rate was calculated from the first treatment date to the date of death within five years or termination within five years. Overall survival (OS) was defined as the time from diagnosis to follow-up death or study termination. Disease-free survival (DFS) is defined as the time from the beginning of randomization to disease recurrence or death due to disease progression. Descriptive analyses of patient characteristics, clinical features, and outcomes were conducted. Calculate the survival time and survival rate and draw the survival curve, and the log-rank test in Kaplan-Meier analysis was used to compare the survival of different categories of patients. Any prognostic factor that was significant in the univariate analysis was selected and included in the multivariate analysis, which was performed using a Cox regression model. After the multivariate Cox analysis, factors with significant differences could be defined as independent prognostic factors. The two-tailed *P* value less than 0.05 indicated a significant difference. All statistical analyses were performed using the SPSS software version 19.0 for Windows (IBM Corp, Armonk, NY, USA).

## 3. Results

### 3.1. Patients and Clinical Baseline Characteristics

One hundred and nineteen qualified patients were retrieved. The demographic and clinicopathological characteristics are shown in Table 1. The flow chart of patient screening in the study is shown in Figure 1. There were 69 men and 50 women included in the analysis with a median age of 60.53 years (ranging from 37 to 78 years). Most of the tumors are located in the middle of the esophagus (78.15%). For TNM stage, the IIb stage (32.77%) and ≥IIIb stage (35.29%) were the main stage. The treatment methods involved in this study included surgery alone (65 cases, 54.62%), surgery combined with postoperative chemotherapy (41 cases, 34.45%), and surgery combined with postoperative chemoradiotherapy (13 cases, 10.93%). Postoperative pathology confirmed that 66 cases (55.46%) were positive for lymph node metastasis.

### 3.2. TNM Stage, T Stage, and Lymph Node Metastasis

To explore the relationship between survival rate of patients and clinicopathological features, several factors were screened, such as gender, age, tumor location, TNM stage, lymph node metastasis, pathological type, and treatment mode, and then, the correlation was analyzed in turn. The median survival time of enrolled patients was 27 months (3-100 months). As shown in Table 2, univariate analysis showed that the median survival time of 53 patients without lymph node metastasis was 48 months, and that of 66 patients with lymph node metastasis was 19 months. Log-rank test showed that the median survival time of patients with different pN stages was significantly different (*P* < 0.05). The median survival time of patients with different pT stages was 38 months, 36 months, 19 months, and 8 months, with significant difference (*P* < 0.05). In pTNM stage, the median survival time of patients with stage I-IIb was 38 months, and that of patients with ≥IIIa stage was 19 months, the difference was statistically significant (*P* < 0.05). The median survival time of patients who received postoperative adjuvant chemotherapy was 36 months, while that of patients who received simple surgery was 21 months, but there was no statistical difference (*P* > 0.05).

### 3.3. Lymph Node Metastasis and Treatment Scheme

According to TNM stage, patients were divided into two subgroups, ≤IIb as a subgroup and ≥IIIA as another subgroup; then, Cox multivariate analysis was performed, respectively. From Table 3, we can find that lymph node metastasis (95% CI: 2.098–34.545; *P* < 0.05) and whether received adjuvant treatment (95% CI: 0.076–1.712; *P* < 0.05) can be used as independent factors to affect the overall survival time of patients with stage I-IIb. However, for patients with stage IIIa and above, there are no significant factors affecting their OS (*P* > 0.05) (Table 4).

To investigate the effect of survival time on patients with esophageal small-cell carcinoma, we performed a Kaplan-Meier analysis. Based on the stratified data, it was observed that TNM staging did not predict 5-year survival in isolated esophageal small-cell carcinoma (*P* = 0.057) (Figure 2(a)). The results also showed that DFS in PSCCE patients was not predictive (*P* = 0.059) (Figure 2(b)).

## 4. Discussion

PSCCE is a malignant tumor with strong invasiveness, high occultity, and easy metastasis, which lacks early symptoms. Patients often seek medical attention for dysphagia, obstruction, and/or frequent vomiting. Weight loss is the main symptom, but it is often diagnosed at an advanced stage [14]. This was also confirmed by the fact that in the majority of patients in this study, postoperative pathology was reported as stage IIb or above (83.19%). This situation leads to a significant reduction in the clinical therapeutic efficacy as well as the quality of life of patients. This study showed that PSCCE mostly occurred in the middle and lower thoracic esophagus (91.60%), which was consistent with previous studies [8, 15, 16].

Another feature of PSCCE is its markedly poor prognosis, so our study of possible underlying factors that might influence OS in patients with this disease helps to explore its survival characteristics. Tumor staging is very useful in determining optimal treatment options; however, due to the low incidence of PSCCE, no specific staging system has been assigned for PSCCE. The most commonly used staging systems today are the American Joint Commission on Cancer (AJCC) staging system [13] and the Veteran's Administration Lung Study Group staging system (VALSG) [17]. Many studies have studied the disease through two staging systems at the same time, which is undoubtedly more comprehensive and also provides ideas for our further research methods. As the AJCC staging system based on TNM staging is widely used in clinical assessment of patient survival, whether its predictive ability is reliable remains controversial. A study of 64 patients showed that stage T was an independent prognostic factor [16], and univariate analysis in this study also showed such results. It seems to be a proven fact that lymph node metastasis (stage N) can affect the prognosis of patients; after all, there are so many research data to provide theoretical support. Li et al. recently demonstrated that regional lymph node staging is an independent prognostic factor for patients with PSCCE. Their results showed that the MST at stage N0 was longer than that at stage N1, N2, and N3 (22.5 versus 22.2 versus 10.7 versus 9.7 months, respectively; *P* < 0.001), and patients with limited lymph node metastasis have a good prognosis [18]. Xu and his colleagues also showed that N0 patients had longer MST than N1, N2, or N3 patients (39.0 versus 28.0 versus 20.0 versus 14.0 months, respectively; *P* < 0.001) by univariate analysis and Cox regression analysis [8]. Situ et al. reported that the presence of multiple regional lymph node metastases was associated with poorer prognosis [19]. In addition, there are more data to support this conclusion [20–22]. Our univariate analysis showed that the median OS (48 months) of patients with negative lymph node metastasis was significantly higher than that of patients with positive lymph node metastasis (19 months), suggesting that PSCCE can change OS through lymph node metastasis, thereby affecting the prognosis of patients.

In the Cox multivariate analysis, our research group innovatively divided patients into two different subgroups according to T stage for analysis, so as to explore whether possible independent factors can affect different stages of disease progression and what kind of influence they have. We found that for the early and middle stage patients (stage I-IIb), lymph node metastasis and treatment scheme were important factors affecting OS in patients with PSCCE. Nevertheless, for intermediate and advanced patients at stage IIIa and above, those factors cannot independently affect patient survival, even if lymph node metastasis is present. This is a new point of view. However, the median OS (19 m) of patients with stage ≥IIIa was significantly shorter than that of patients with stage ≤IIb (38 m). Based on clinical experience, we speculate that the reason for this result may be that patients with advanced disease have a longer course of disease, are often accompanied by multiple lymph node metastases or even distant metastases, have poor response to various treatments, and have poor therapeutic effects. Therefore, treatment is difficult to effectively delay disease progression and prolong survival. However, these still require more data and further studies to verify.

With the advancement of surgical techniques and the consensus of clinical experience, esophagectomy has gradually become the main treatment method for PSCCE. All patients included in the study have received appropriate surgical treatments according to their respective conditions. As a protective factor, surgery can reduce the specific mortality by nearly 76% [23], but whether postoperative adjuvant treatment can benefit patients remains to be determined. A stratified analysis of 152 patients by Xu et al. found that postoperative adjuvant therapy could not improve the OS (*P* = 0.522) or DFS (*P* = 0.368) [8]. However, Chen et al. pointed out that compared with surgery alone, postoperative chemotherapy can improve the survival rate (13 versus 6.1 months, *P* = 0.003), while increasing radiotherapy can also improve the survival rate to some extent (16.8 versus 9.5 months, *P* = 0.076) [21]. Some studies have also shown that PSCCE should be treated as a systemic disease, and postoperative chemotherapy and radiotherapy should be used as routine treatments [24, 25]. According to the results of this study, the treatment modality could exist as an independent factor affecting OS in patients with stage I-IIb, but it was not significant in patients with stage ≥IIIa. In this regard, some studies have also shown that chemoradiotherapy is the main method to improve the survival rate of patients with stage III or above [26, 27].

To date, most studies have shown OS as the primary endpoint. Since TNM stage affects survival outcomes at OS discontinuation, we performed a survival analysis using Kaplan-Meier to explore its effect on five-year survival time and DFS. Unfortunately, our results suggest that TNM staging does not predict five-year OS or DFS in PSECC.

## 5. Conclusions

PSCCE usually occurs in the middle and lower esophagus, with a high degree of malignancy and poor prognosis. Our study showed that TNM staging, T staging, and lymph node metastasis are related to the survival of patients. Negative lymph node metastasis and treatment are favorable independent prognostic factors for patients with stage I-IIb of PSCCE. Therefore, we suggest that appropriate adjuvant therapy should be added to these patients after surgery.

## Figures and Tables

**Figure 1:** Patient screening flow chart. A total of 119 patients with PSCCE were included in the study.

**Figure 2:** Kaplan-Meier survival curve. (a) Five-year survival for patients at different TNM stages; (b) DFS for patients at different TNM stages. DFS: disease-free survival.

**Table 1:** Baseline characteristics of PSCCE patients.

	Number	Rate
Gender		
Male	69	57.98
Female	50	42.02
Age (year, mean ± SD)	60.53 ± 8.35	
Tumor local		
Upper	10	8.4
Middle	93	78.15
Lower	16	13.45
pTNM stage		
I-IIa	20	16.81
IIb	39	32.77
IIIa	18	15.13
≥IIIb	42	35.29
Lymph node metastasis		
Negative	53	44.54
Positive	66	55.46
Therapy		
Surgery only	65	54.62
Surgery with chemotherapy	41	34.45
Surgery with chemoradiotherapy	13	10.93

PSCCE: primary small-cell carcinoma of esophagus; T: tumor; N: regional lymph node; M: metastasis; SD: standard deviation.

**Table 2:** Univariate analysis of factors affecting OS of patients with PSCCE.

	Number	Median OS (m)	*χ* ^2^	*P* value
Gender			0.001	0.97
Male	69	36		
Female	50	23		
Age (year)			1.277	0.259
≤60	68	32		
>60	51	19		
Tumor local			1.509	0.47
Upper	10	23		
Middle	93	26		
Lower	16	20		
pTNM stage			7.23	0.007
I-IIb	59	38		
≥IIIa	60	19		
pT stage			7.844	0.049
1	33	38		
2	35	36		
3	50	19		
4	1	8		
Lymph node metastasis			8.32	0.004
Negative	53	48		
Positive	66	19		
Therapy			3.31	0.191
Surgery only	65	21		
Surgery with chemotherapy	41	36	3.272	0.07
Surgery with chemoradiotherapy	13	19		

OS: overall survival; T: tumor; N: regional lymph node; M: metastasis.

**Table 3:** Cox multivariate analysis of factors affecting OS in ≦IIb stage.

	*B*	SE	*χ* ^2^	df	*P* value	Exp(*B*)	95% CI for Exp(*B*)
Gender	0.82	0.59	1.93	1	0.16	2.27	0.714~7.226
T stage	0.36	0.28	1.61	1	0.21	1.43	0.822~2.488
N metastasis	2.14	0.72	8.98	1	0.003	8.51	2.098~34.545
Biopsy pathological diagnosis	-0.54	0.55	0.97	1	0.33	0.58	0.198~1.712
Therapy mode	-1.54	0.53	8.47	1	0.004	0.214	0.076~7.226

**Table 4:** Cox multivariate analysis of factors affecting OS in ≥IIIa stage.

	*B*	SE	*χ* ^2^	df	*P* value	Exp(*B*)	95% CI for Exp(*B*)
Gender	-0.03	0.41	0.004	1	0.948	0.974	0.44~2.156
T stage	-0.01	0.374	0.001	1	0.979	0.99	0.475~2.062
Biopsy pathological diagnosis	-0.31	0.373	0.668	1	0.414	0.737	0.355~1.531
Therapy mode	-0.01	0.237	0.001	1	0.981	0.994	0.625~1.582

OS: overall survival; *B*: regression coefficient; SE: standard error; CI: confidence interval; T: tumor.

## Data Availability

The data used to support the findings of this study were supplied by the Institutional Ethnics Committee of the Fourth Hospital of Hebei Medical University under license and so cannot be made freely available. Requests for access to these data should be made to Dr. Jidong Zhao, e-mail: zjd2016@hebmu.edu.cn.

## References

[1] McKeown F. (1952). Oat-cell carcinoma of the oesophagus. *The Journal of Pathology and Bacteriology*.

[2] Miao H., Li R., Chen D., Hu J., Chen Y., Wen Z. (2021). Survival outcomes and prognostic factors of primary small cell carcinoma of the esophagus. *Journal of Thoracic Disease*.

[3] Xiao Q., Xiao H., Ouyang S., Tang J., Zhang B., Wang H. (2019). Primary small cell carcinoma of the esophagus: comparison between a Chinese cohort and Surveillance, Epidemiology, and End Results (SEER) data. *Cancer Medicine*.

[4] Cicin I., Karagol H., Uzunoglu S. (2007). Extrapulmonary small cell carcinoma compared with small cell lung carcinoma: a retrospective single-center study. *Cancer*.

[5] Meng M. B., Zaorsky N. G., Jiang C. (2013). Radiotherapy and chemotherapy are associated with improved outcomes over surgery and chemotherapy in the management of limited-stage small cell esophageal carcinoma. *Radiotherapy and Oncology*.

[6] Wong A. T., Shao M., Rineer J., Osborn V., Schwartz D., Schreiber D. (2017). Treatment and survival outcomes of small cell carcinoma of the esophagus: an analysis of the National Cancer Data Base. *Diseases of the Esophagus*.

[7] Tao H., Li F., Wang J. (2015). Management of treatment-naïve limited-stage small cell esophagus carcinoma. *Saudi Medical Journal*.

[8] Xu L., Li Y., Liu X. (2017). Treatment strategies and prognostic factors of limited-stage primary small cell carcinoma of the esophagus. *Journal of Thoracic Oncology*.

[9] Nayal B., Vasudevan G., Rao A. C. K. (2015). Primary small cell carcinoma of the esophagus-an eight year retrospective study. *Journal of Clinical and Diagnostic Research*.

[10] Xie M. R., Xu S. B., Sun X. H. (2015). Role of surgery in the management and prognosis of limited-stage small cell carcinoma of the esophagus. *Diseases of the Esophagus*.

[11] Kojima T., Doi T. (2017). Immunotherapy for esophageal squamous cell carcinoma. *Current Oncology Reports*.

[12] Bagnardi V., Rota M., Botteri E. (2015). Alcohol consumption and site-specific cancer risk: a comprehensive dose-response meta-analysis. *British Journal of Cancer*.

[13] Rice T. W., Rusch V. W., Ishwaran H., Blackstone E. H. (2010). Cancer of the esophagus and esophagogastric junction: datadriven staging for the seventh edition of the American Joint Committee on Cancer/International Union Against Cancer Cancer Staging Manuals. *Cancer*.

[14] Wu Y. H., Zhang K., Chen H. G., Wu W. B., Li X. J., Zhang J. (2021). Primary small cell esophageal carcinoma, chemotherapy sequential immunotherapy: a case report. *World Journal of Clinical Cases*.

[15] Cai G., Wang J., Zou B. (2021). Preoperative chemotherapy for limited-stage small cell carcinoma of the esophagus. *The Annals of Thoracic Surgery*.

[16] Zhu Y., Qiu B., Liu H. (2014). Primary small cell carcinoma of the esophagus: review of 64 cases from a single institution. *Diseases of the Esophagus*.

[17] Micke P., Faldum A., Metz T. (2002). Staging small cell lung cancer: Veterans Administration Lung Study Group versus International Association for the Study of Lung Cancer--what limits limited disease?. *Lung Cancer*.

[18] Li R., Yang Z., Shao F. (2021). Multi-omics profiling of primary small cell carcinoma of the esophagus reveals RB1 disruption and additional molecular subtypes. *Nature Communications*.

[19] Situ D., Lin Y., Long H. (2013). Surgical treatment for limited-stage primary small cell cancer of the esophagus. *The Annals of Thoracic Surgery*.

[20] Zhang B. H., Yang W. J., Zhao L., He J., Wang Y. G., Zhang H. T. (2012). Surgical treatment and prognostic analysis of 109 patients with primary esophageal small cell carcinoma. *Zhonghua Zhong Liu Za Zhi*.

[21] Chen W. W., Wang F., Chen S. (2014). Detailed analysis of prognostic factors in primary esophageal small cell carcinoma. *The Annals of Thoracic Surgery*.

[22] Sun K. L., He J., Cheng G. Y., Chai L.-x. (2007). Management of primary small cell carcinoma of the esophagus. *Chinese Medical Journal*.

[23] Zhang G., Wu B., Wang X., Li J. (2019). A competing-risks nomogram and recursive partitioning analysis for cause-specific mortality in patients with esophageal neuroendocrine carcinoma. *Diseases of the Esophagus*.

[24] Zhao K., Huang Z., Si Y., Sun L., Yu J., Meng X. (2021). Use of chemoradiotherapy as a treatment option for patients with limited-stage primary small cell carcinoma of the esophagus. *Cancer Management and Research*.

[25] Murakami K., Akutsu Y., Miyazawa Y. (2011). A case of small-cell esophageal cancer with chronic renal failure undergoing hemodialysis safely treated with cisplatin and etoposide. *Esophagus*.

[26] Shapiro J., van Lanschot J. J. B., Hulshof M. C. C. M. (2015). Neoadjuvant chemoradiotherapy plus surgery versus surgery alone for oesophageal or junctional cancer (CROSS): long-term results of a randomised controlled trial. *The Lancet Oncology*.

[27] Hou X., Wei J.-C., Wu J.-X. (2013). Multidisciplinary modalities achieve encouraging long-term survival in resectable limited-disease esophageal small cell carcinoma. *PLoS One*.

